# Shared Molecular Mechanisms between Alzheimer's Disease and Periodontitis Revealed by Transcriptomic Analysis

**DOI:** 10.1155/2021/6633563

**Published:** 2021-04-01

**Authors:** Jieqi Jin, Mengkai Guang, Anthony Chukwunonso Ogbuehi, Simin Li, Kai Zhang, Yihong Ma, Aneesha Acharya, Bihan Guo, Zongwu Peng, Xiangqiong Liu, Yupei Deng, Zhaobi Fang, Xiongjie Zhu, Shiting Hua, Cong Li, Rainer Haak, Dirk Ziebolz, Gerhard Schmalz, Lei Liu, Baohua Xu, Xiaofeng Huang

**Affiliations:** ^1^Department of Stomatology, Beijing Friendship Hospital, Capital Medical University, Beijing 100050, China; ^2^Department of Stomatology, China-Japan Friendship Hospital, Beijing 100029, China; ^3^Department of Physics, University of Münster, Wilhelm-Klemm-Str. 9, 48149 Münster, Germany; ^4^Department of Cariology, Endodontology and Periodontology, University Leipzig, Liebigstr. 12, Leipzig 04103, Germany; ^5^Department of Neurology, Graduate School of Medical Sciences, Faculty of Life Sciences, Kumamoto University, Kumamoto, Japan; ^6^Dr. D Y Patil Dental College and Hospital, Dr D Y Patil Vidyapeeth, Pimpri, Pune, India; ^7^Faculty of Electrical Engineering, Information Technology, and Physics, University Braunschweig, Hans-Sommer-Str. 66, Braunschweig 38106, Germany; ^8^Laboratory of Molecular Cell Biology, Beijing Tibetan Hospital, China Tibetology Research Center, 218 Anwaixiaoguanbeili Street, Chaoyang, Beijing 100029, China; ^9^Zhujiang Hospital, Southern Medical University, Guangzhou 510282, China; ^10^Department of Neurology, Shandong Provincial Third Hospital, Cheeloo College of Medicine, Shandong University, Jinan, 10091 Shandong Province, China

## Abstract

**Objective:**

To investigate the genetic crosstalk mechanisms that link periodontitis and Alzheimer's disease (AD).

**Background:**

Periodontitis, a common oral infectious disease, is associated with Alzheimer's disease (AD) and considered a putative contributory factor to its progression. However, a comprehensive investigation of potential shared genetic mechanisms between these diseases has not yet been reported.

**Methods:**

Gene expression datasets related to periodontitis were downloaded from the Gene Expression Omnibus (GEO) database, and differential expression analysis was performed to identify differentially expressed genes (DEGs). Genes associated with AD were downloaded from the DisGeNET database. Overlapping genes among the DEGs in periodontitis and the AD-related genes were defined as crosstalk genes between periodontitis and AD. The Boruta algorithm was applied to perform feature selection from these crosstalk genes, and representative crosstalk genes were thus obtained. In addition, a support vector machine (SVM) model was constructed by using the scikit-learn algorithm in Python. Next, the crosstalk gene-TF network and crosstalk gene-DEP (differentially expressed pathway) network were each constructed. As a final step, shared genes among the crosstalk genes and periodontitis-related genes in DisGeNET were identified and denoted as the core crosstalk genes.

**Results:**

Four datasets (GSE23586, GSE16134, GSE10334, and GSE79705) pertaining to periodontitis were included in the analysis. A total of 48 representative crosstalk genes were identified by using the Boruta algorithm. Three TFs (FOS, MEF2C, and USF2) and several pathways (i.e., JAK-STAT, MAPK, NF-kappa B, and natural killer cell-mediated cytotoxicity) were identified as regulators of these crosstalk genes. Among these 48 crosstalk genes and the chronic periodontitis-related genes in DisGeNET, C4A, C4B, CXCL12, FCGR3A, IL1B, and MMP3 were shared and identified as the most pivotal candidate links between periodontitis and AD.

**Conclusions:**

Exploration of available transcriptomic datasets revealed C4A, C4B, CXCL12, FCGR3A, IL1B, and MMP3 as the top candidate molecular linkage genes between periodontitis and AD.

## 1. Introduction

An association between periodontitis and Alzheimer's disease (AD) has been demonstrated, and periodontitis reportedly confers risk for the incidence and progression of Alzheimer's disease (AD) [1, 2]. Alzheimer's disease is a neurodegenerative disease characterized by the formation of amyloid-*β* peptide (A*β*P) plaques and intraneuronal neurofibrillary tangles (NFTs), which drives neuroinflammation in the brain [3]. Periodontitis, a chronic, immunoinflammatory disease affecting supporting structures of teeth, is multifactorial in nature, driven by polymicrobial dysbiosis and unfavorable shifts in the plaque biofilm composition, which disrupts the host-microbial homeostasis [4, 5]. Inflammation is considered the key connecting link between both these diseases [6]. Two purported mechanistic links have been highlighted. First, proinflammatory mediators including specific cytokines or chemokines in the periodontal milieu that enter systemic circulation impose a systemic inflammatory burden, propagating inflammatory responses by microglial cells in the brain [6]. Second, periodontal pathogens may directly enter the brain via blood circulation or peripheral nerves, as evidenced by the discovery of the keystone periodontal pathogen *Porphyromonas gingivalis* (Pg) in AD patients' brains [7, 8].

At the same time, genetic susceptibility and gene dysregulation have been identified in the context of both AD and periodontitis. In AD, frequently reported dysregulated genes include amyloid-beta precursor protein (APP), presenilin 1 (PSEN1), and presenilin 2 (PSEN2), apolipoproteins, and lipid homeostasis, genes involved in endocytosis, and membrane-spanning 4 (MS4) family [9]. In periodontitis, aberrant genes highlighted include interleukin-1, interleukin-6, interleukin-10, transforming growth factor-beta (TGF-*β*), tumor necrosis factor-*α* (TNF-*α*), interferon-gamma (IFN-*γ*), and matrix metalloproteinases (MMPs) among others [10]. It is plausible that gene dysregulation in periodontitis could contribute to its association with AD, and crosstalk genes may biologically link AD and periodontitis serving as either shared susceptibility factors or molecular links.

Here, we designed a bioinformatic study of existing experimental datasets to understand putative molecular links between periodontitis and Alzheimer's disease by identifying crosstalk genes, transcription factors, and signaling pathways involved in both disorders. The molecular mechanisms identified through this approach could suggest potential therapeutic targets particularly relevant to drug development and personalized medicine approaches.

## 2. Materials and Methods

### 2.1. Study Design

Figure 1 depicts a flowchart outlining the study workflow. DEGs dysregulated in periodontitis- and AD-related genes were obtained from the GEO database and DisGeNET database, respectively. Crosstalk genes linking periodontitis and AD were identified as the AD-related genes that overlapped with significantly up- or downregulated DEGs in periodontitis. Thereafter, feature selection from the crosstalk genes was performed using a conventional recursive feature elimination (RFE) algorithm and the Boruta algorithm. The crosstalk genes obtained by feature selection were used to construct two networks to identify the transcription factors and the differentially expressed pathways that target these crosstalk genes. In the next step, “core” crosstalk genes were identified as the crosstalk genes obtained by feature selection that were overlapping with chronic periodontitis-related genes in the DisGeNET database.

### 2.2. Procurement of Periodontitis-Related Datasets

Sample-matched whole-genome gene expression datasets from periodontitis were sourced and downloaded from the NCBI Gene Expression Omnibus (GEO). The eligibility criteria for these datasets were as follows: datasets that included established periodontitis samples as the experimental group and healthy gingival samples as the control group, where periodontitis was defined based in accordance with the case definition presented in the 2017 World Workshop: (1) interdental CAL detectable at ≥2 nonadjacent teeth or (2) buccal or oral CAL ≥ 3 mm with pocketing >3 mm detectable at ≥2 teeth [11].

### 2.3. Differential Gene Expression Analysis

Differential gene expression analysis of periodontitis-related datasets was carried out using the Linear Models for Microarray (limma) package [12] in the R project (version 3.0.1, http://www.r-project.org/) [13]. Three such datasets, GSE23586, GSE16134, and GSE10334, were sourced and analyzed. Genes with *p* value < 0.05 and ∣logFC (fold change) | ≥1 were regarded as significant differentially expressed genes (DEGs). For another dataset, GSE79705, the screening range of DEGs was broadened by extending the thresholds and settings to *p* value < 0.05 and ∣logFC | >0 as DEGs.

Next, a Venn diagram (http://bioinformatics.psb.ugent.be/webtools/Venn/) was drawn to identify shared genes within the DEGs identified from the four datasets. The common up/downregulated DEGs in four datasets were used for the following analyses, and DEGs that were not common to all the datasets were excluded.

### 2.4. Functional Enrichment Analysis

Functional enrichment analysis of up/downregulated periodontitis-related DEGs was performed with DAVID (Database for Annotation, Visualization and Integrated Discovery, v6.8) [14, 15]. *p* < 0.05 was set as the threshold. GO (Gene Ontology) and pathway enrichment analysis of the identified DEGs was performed [16, 17].

### 2.5. Construction of the Protein-Protein Interaction Network of Periodontitis-Related DEGs

280,826 PPI (protein-protein interaction) pairs including 19,610 genes were downloaded from HPRD (Human Protein Reference Database) [18], BioGRID (Biological General Repository for Interaction Datasets) [19], DIP (Database of Interacting Proteins) [20], MINT (Molecular INTeraction database) [21], PINA (Protein Interaction Network Analysis) [22], InnateDB (a knowledge resource for innate immunity interactions and pathways) [23], and INstruct (3D protein interactome networks with structural resolution) [24]. The Cytoscape platform was used to visualize the network derived from PPI pairs of DEGs and conduct a topological analysis [25].

### 2.6. Identification of Crosstalk Genes and Construction of the Crosstalk Gene-Related PPI Network

AD-related genes were downloaded from the DisGeNET database [26]. The AD-related genes that overlapped with the up- and downregulated periodontitis-related DEGs were identified. These overlapping genes were regarded as “crosstalk” genes linking AD and periodontitis and further used for constructing a crosstalk gene-related PPI network. The crosstalk gene-related PPI network consisted of four types of nodes, namely, (1) DEGs dysregulated in periodontitis (not related to AD), (2) crosstalk genes or AD-related genes which were also DEGs dysregulated in periodontitis, (3) AD-related genes (not dysregulated in periodontitis), and (4) other genes (neither related to AD nor dysregulated in periodontitis).

### 2.7. Feature Selection from Crosstalk Genes

Since GSE16134 had the largest sample size among the periodontitis-related datasets, it was used as the test set. The other three datasets (GSE23586, GSE10334, and GSE79705) were used as validation sets. Firstly, expression values of the crosstalk genes (identified in the previous step) from GSE16134 were used as input for the Boruta algorithm in the R project [27] and the conventional recursive feature elimination (RFE) algorithm [28] and feature selection was performed. Each gene was regarded as a feature.

### 2.8. Support Vector Machine (SVM) Modeling Using Feature-Selected Crosstalk Genes

The expression values in GSE16134 and GSE10334 were scale-standardized. Next, it was examined if the crosstalk genes obtained by feature selection were found in the four periodontitis-related datasets (i.e., GSE23586, GSE16134, GSE10334, and GSE79705). The gene expression values of these feature selection-obtained crosstalk genes were extracted from these datasets. If the number of expression profile genes in a certain dataset after extraction was lower than the number of feature selection-obtained crosstalk genes, the expression values of the missing genes were considered missing values and represented by the NA symbol. The missing values were processed by using the DMwR package [29] in R, and the *K*-Nearest Neighbors (KNN) algorithm was used to impute these missing values (NA) in that dataset. By imputing these missing values, all the four periodontitis-related datasets presented all the feature selection-obtained crosstalk genes. Thereafter, the scikit-learn package [30] was used to perform a grid search, and the best hyperparameters of a support vector machine (SVM) model were found by using 5-fold cross-validation (CV) [31]. A SVM classifier model was established by using data from GSE16134 as the training set and test set, where the samples of the GSE16134 dataset were split into 60% : 40% for the training set and test set, respectively. Data from the other three datasets (GSE23586, GSE10334, and GSE79705) were used as the validation set. The decision function method was used to obtain the score for each sample. Next, receiver operating characteristic (ROC) curves for the four datasets were generated by using the pROC package and displayed using the ggplot2 package in R.

### 2.9. Targeting Relationships between Transcription Factors (TFs) and Crosstalk Genes

Transcription factor- (TF-) target gene regulation pairs were obtained and downloaded from TRRUST [32], cGRNB [33], HTRIdb [34], ORTI [35], and TRANSFAC [36] databases. The TF-target gene interaction pairs corresponding to the feature selection-obtained crosstalk genes were extracted and used for constructing a TF-target gene interaction network with visualization using Cytoscape software [37].

### 2.10. Pathway Analysis of the Crosstalk Genes

Human data describing relationships between signaling pathways and genes were downloaded from the KEGG database, and all pathways related to the feature selection-obtained crosstalk genes were extracted. The expression levels of these crosstalk gene-related pathways were plotted as a heatmap, and differential expression analysis was performed and applied to the four periodontitis-related datasets to identify the DEPs (differentially expressed pathways) using the R package limma. For the three datasets (GSE23586, GSE16134, and GSE79705), the pathways with *p* value < 0.05 and ∣logFC | ≥1 were regarded as differentially expressed pathways (DEPs), while for the dataset GSE79705, the pathways with *p* value < 0.05 and ∣log FC | >0 were regarded as DEPs.

### 2.11. Classification Performance of the Core Crosstalk Genes

The genes related to periodontitis were downloaded from the DisGeNET database [26]. The overlap between the periodontitis-related genes obtained from the DisGeNET database and the feature selection-obtained crosstalk genes was analyzed, and the overlapping genes were termed core crosstalk genes. The corresponding expression values of these overlapping genes in the four periodontitis-related datasets were obtained, and ROC curves were drawn.

## 3. Results

### 3.1. Included Periodontitis-Related Datasets

Four datasets pertaining to periodontitis (i.e., GSE23586, GSE16134, GSE10334, and GSE79705) were included and analyzed.  Table 1 provides key details regarding the included datasets.

### 3.2. Identification of Periodontitis-Related DEGs and Their Functions

Table 2 shows the number of up- and downregulated DEGs that were identified in each of the four datasets.  Figure 2 depicts a Venn diagram showing the overlap of DEGs identified from the four datasets. A total of 816 DEGs including 405 upregulated genes and 411 downregulated genes were used for the following analyses.  Figure 3 shows the biological processes and signaling pathways in which the up- and downregulated DEGs were significantly enriched.

### 3.3. The Hub Genes Identified by the Periodontitis-Related PPI Network

Figure 4 depicts a PPI network based on the periodontitis-related DEGs, and Table 3 shows the topological characteristics of the top 30 nodes in the PPI network. As seen in Table 3, several genes with the highest degree were identified as hub genes. These upregulated DEGs included SMAD3, TRIM27, VIM, YWHAH, and FOS, and downregulated DEGs included MYC, HSPB1, DDB1, RPS3, KAT5, SMARCA4, RPL13, and PLCG1.

### 3.4. Crosstalk Genes Bridging Alzheimer's Disease and Periodontitis

In total, 51 upregulated crosstalk genes and 41 downregulated crosstalk genes were identified and are listed in Table 4. The crosstalk gene-related PPI network as shown in Figure 5 consisted of 3496 nodes and 5141 edges. The topological characteristics of the top 30 nodes in this network are presented in Table 5. Hub crosstalk genes with the highest degree included MYC, HSPB1, VIM, KAT5, RPL13, FOS, and CDH1.

### 3.5. Crosstalk Genes Obtained by Feature Selection

A total of 48 crosstalk genes were selected by using the Boruta algorithm (Figure 6(a)). In addition, 62 crosstalk genes were selected by using the RFE algorithm (Figure 6(b)). All 48 genes obtained by using the Boruta algorithm were included in the 62 genes obtained by the RFE algorithm, indicating that this 48-gene set was representative of the characteristics of all 92 crosstalk genes.

### 3.6. Classification Accuracy Using the Feature Selection-Obtained Crosstalk Genes

The 48 genes obtained by SVM feature selection were not shown in all of the four periodontitis-related datasets. The gene expression profiles of GSE16134 and GSE10334 included all of the 48 crosstalk genes, whereas GSE23586 included 44 crosstalk genes and GSE79705 included 45 crosstalk genes. The classification performance of these 48 crosstalk genes for the four datasets is shown in Table 6. For the test set GSE16134 and the validation set GSE10334, the accuracy performance was high at 91.94% and 88.26%, respectively. By comparison, the performance for the other two datasets GSE23586 and GSE79705 was low at 50% and 66.66%, respectively.

### 3.7. ROC Curves for the Four Periodontitis-Related Datasets

As shown in Figure 7, the AUC (area under the curve) values for the GSE16134 test set and the GSE10334 validation set were high at 95.77% and 90.53%, respectively, congruent with the results in Table 6. It was thus inferred that the classifier performance was adequate only when the sample sizes of the validation sets were similar to those of the training and test datasets, and therefore, poor performance was noted for GSE23586 and GSE79705 having much lower sample numbers.

### 3.8. The Identification of Transcription Factors Regulating the Crosstalk Genes

As shown in Figure 8, the TF-crosstalk gene target network consisted of 388 nodes and 1178 edges. Several transcription factors which were also DEGs played critical roles by regulating the most number of crosstalk genes, for example, FOS, MEF2C, and USF2 (Table 7).

### 3.9. Signaling Pathways Enriched in the Crosstalk Genes

From the 48 feature selection-obtained crosstalk genes, 37 crosstalk genes were found among gene-pathway interaction pair data in the KEGG database. 137 KEGG pathways corresponded to these 37 crosstalk genes.  Figure 9 shows the expression values of these 137 pathways in the four periodontitis-related datasets.

The numbers of crosstalk gene-related DEPs obtained from each of the four periodontitis-related datasets are listed in Table 8. The interaction relationships between crosstalk genes and DEPs are depicted in Figure 10, showing that several DEPs were dysregulated in at least two datasets, including cytokine-related pathways (cytokine-cytokine receptor interaction, chemokine, and IL-17), immune cell-related pathways (T cell receptor, B cell receptor, Th1 and Th2 cell differentiation, Th17 cell differentiation, natural killer cell-mediated cytotoxicity, and osteoclast differentiation), JAK-STAT signaling, NOD-like receptor signaling, MAPK signaling, Toll-like receptor signaling, NF-kappa B signaling, and C-type lectin receptor signaling.

### 3.10. The Identification of Core Crosstalk Genes

Among the 48 feature selection-obtained crosstalk genes and periodontitis-related genes in the DisGeNET database, 12 common genes were identified as core crosstalk genes including C3, C4A, C4B, CXCL12, FCGR3A, FCGR3B, HSPB1, IL1B, MME, MMP3, PLAT, and VEGFA (Table 9). Among these 12 genes, 6 genes, C4A, C4B, CXCL12, FCGR3A, IL1B, and MMP3, were found associated with chronic periodontitis.

Figure 11 shows ROC curves for the 6 chronic periodontitis-related genes for each of the four datasets. An AUC value of more than 80% was presented by three genes, C4A, C4B, and CXCL12, for the dataset GSE10334, 5 genes, C4A, C4B, CXCL12, FCGR3A, and IL1B, for GSE16134, 3 genes, CXCL12, IL1B, and MMP3, for GSE23586, and all 6 genes for GSE79705. The 3 genes, C4A, C4B, and CXCL1, had the highest classification accuracy when the datasets with small samples (GSE23586 and GSE79705) were not considered.

## 4. Discussion

The present study addressed shared genetic mechanisms and molecular links between periodontitis and Alzheimer's diseases by identifying gene expression, signaling pathways, and TFs that were most robustly associated with both these diseases. These findings are largely substantiated by preexisting experimental data.

Six genes C4A, C4B, CXCL12, FCGR3A, IL1B, and MMP3 were identified as the most significant crosstalk genes linking chronic periodontitis and Alzheimer's disease. C4B and C4A, respectively, encode the basic and acidic forms of the complement factor 4, and C4 gene deficiency has been noted to predispose the development of severe chronic periodontitis [38]. In AD, the expression levels of C4 mRNA were shown to be 3.27-fold increased in temporal cortex samples as compared to controls [39]. The CXCL12 (C-X-C motif chemokine ligand 12) gene is the ligand of the C-X-C motif chemokine receptor 4 (CXCR4). CXCL12 expression in the gingival crevicular fluid of periodontitis patients was shown to be significantly higher than that of healthy subjects, suggesting that it might play a role in enhancing neutrophil migration and further the progression of periodontitis [40]. A decreased level of CXCL12 in Alzheimer's disease has been documented as affecting cognitive function, impairing learning and memory [41]. FCGR3A (Fc fragment of IgG receptor IIIa) encodes a receptor for the Fc portion of immunoglobulin G, and FCGR3A polymorphisms are shown to confer susceptibility to periodontitis in Caucasians [42]. In AD, the Fc gamma receptor (Fc*γ*R) was recently found to exacerbate neurodegeneration [43]. Cytokines are considered a primary link between chronic periodontitis and Alzheimer's disease as they can enter systemic circulation through periodontal pockets [6]. The classical proinflammatory cytokine, IL1B, is elevated in periodontitis and can induce resorption of alveolar bone [44]. In AD, IL1B gene polymorphisms are linked to disease susceptibility [45]. MMP3 (matrix metalloproteinase 3) is implicated in the progression of chronic periodontitis and can degrade the periodontal tissue matrix [46]. Elevated brain levels of MMP3 have been associated with the duration of Alzheimer's disease, and it has been found to increase the activity of MMP9, thereby indirectly promoting aggregation and cerebral accumulation of tau deposits [47].

More interestingly, the six genes discussed in the last paragraph were also found to be the molecular crosstalks in linking the peripheral immune system and central nervous system (CNS). It has been well demonstrated that the periodontal disease-evoked peripheral systemic host immune response can aggravate the progression of neuroinflammation and neurodegeneration in Alzheimer's disease by switching the microglia from the primed phenotype to an aggressive proinflammatory phenotype [48, 49]. The immune-inflammatory mediators (e.g., cytokines and chemokines) abundantly expressed during periodontal inflammation can circulate into the bloodstream and travel into the brain by crossing the blood-brain barrier (BBB) and impact the function of CNS [50]. Therefore, the crosstalk between the peripheral immune system and the CNS might be an important mechanism underlying periodontitis, increasing the risk of AD. This paragraph will provide a description regarding the potential role of the six crosstalk genes in linking periodontal disease and AD, especially by means of neuroimmune interaction. For example, the complement components C4A and C4B highly expressed in periodontal disease were found to modulate T cell immune response by stimulating the activation and migration of T cells [51–53]. The migration of T cells enhanced by C4A and C4B might allow T cells to traffic across the BBB and enter the brain. For another example, the chemokine and its receptor-composed system CXCL12/CXCR4-7 system were found to be a significant player of the neuroimmune interface [54]. On the one hand, the chemokine CXCL12 mediated the immune-inflammatory response in CNS by recruiting lymphocytes and macrophages [55]. On the other hand, CXCL12 can lead to neurotoxicity and neurodegenerescence by activating the neuronal survival-associated G protein-activated inward rectifier K(+) (GIRK) [54]. FCGR3A (also named CD16) is essential for the antibody-dependent cellular cytotoxicity (ADCC) mediated by natural killer (NK) cells [56]. The increased cytotoxic activity of NK cells was found to cause the dysregulation of protein kinase C and further led to the cognitive deficits in Alzheimer's disease, indicating the contribution of immunological factors to the dysfunction of CNS [57]. IL1B, which was upregulated in periodontitis and transported through the vascular circulation into the brain, was found to play promoting roles in neuroinflammation by enhancing the expression of leukocyte chemotactic chemokines, cell surface adhesion molecules, cyclooxygenases, and MMPs within the brain parenchyma [58]. Likewise, MMP3 abundantly produced in periodontitis was also found to be associated with neuroinflammation via activating microglial cells, as well as participating in the BBB breakdown through the proteolysis of fibronectin and type IV collagen [59]. Taken together, the six crosstalk genes identified in the present research were well evidenced to be involved in periodontitis-triggered peripheral systemic host immune response caused CNS dysfunction in Alzheimer's disease.

Three transcription factors, FOS, MEF2C, and USF2, were identified as related to the regulation of the crosstalk genes and were also found to be dysregulated in chronic periodontitis. The proto-oncogene FOS (also named C-Fos) was found to be involved in the transcriptional regulation of collagenase and cell proliferation genes in periodontal gingival fibroblasts [60]. In AD, FOS is reported to initiate amyloid-*β*-mediated apoptosis and found to be increased in the hippocampal regions of AD patients [61]. Myocyte-specific enhancer factor 2C (MEF2C) was identified as a critical transcription factor involved in the coexpression network of chronic periodontitis [62]. Genome-wide association studies (GWAS) have shown the linkage between mutation of MEF2C and aging-associated late-onset Alzheimer's disease [63, 64]. Experimentally, a lack of MEF2C expression was shown to exaggerate microglial response and negatively affect brain function [65]. The USF2 (upstream transcription factor 2, C-Fos interacting) transcription factor is reported to enhance osteogenic differentiation of periodontal ligament cells (PDLCs) [66]; however, its involvement in periodontal inflammation has not been reported. In the context of AD, the USF2 gene was shown to regulate the expression of genes Dhcr24, Aplp2, Tia1, Pdrx1, Vdac1, and Syn2, which drive the neuropathological mechanisms [67]. However, a study of Japanese participants found that the single nucleotide polymorphisms of the USF2 gene were not significantly related to the onset of AD [68].

Differentially expressed pathways were identified from the crosstalk gene-pathway network, and several pathways including JAK-STAT, MAPK, NF-kappa B, and natural killer cell-mediated cytotoxicity were found as the most robust differentially expressed pathways in at least two periodontitis datasets. Overall, experimental evidence supports these as linkage mechanisms between periodontitis and AD. The activation of the JAK-STAT pathway induced by the *Porphyromonas gingivalis* lipopolysaccharide (LPS) and nicotine was shown to increase the expression of cyclooxygenase-2 (COX-2), prostaglandin E2 (PGE2), and proinflammatory cytokines in osteoblasts, thus further accelerating periodontitis progression [69, 70]. In AD, the inhibitor of the JAK-STAK pathway is reported as a therapeutic target, and blocking this pathway can protect against neuroinflammation and dopaminergic neurodegeneration [71]. The MAPK pathway is the upstream signaling intermediate to many inflammatory cytokines such as TNF-*α*, IL-1*β*, IL-6, and prostaglandin E2 [72], and the blockage of this pathway could be beneficial for treating inflammatory diseases like chronic periodontitis and AD [73, 74]. The activation of MAPK signaling is noted to promote the production of MMPs and RANKL, leading to osteoclastogenesis and the acceleration of alveolar bone loss [73]. MAPK signaling is also implicated in multiple aspects of the neuropathology of AD, such as promoting neuroinflammation, amyloid-beta toxicity and aggregation, autophagy, and apoptosis [75]. The overexpression of NF-*κ*B signaling plays a pivotal role in periodontitis-associated bone destruction by promoting the differentiation and activation of osteoclasts [76]. The blockade of NF-*κ*B signaling is found to trigger detrimental neural alterations including neuroinflammation, activation of microglia, oxidative stress-related complications, and apoptosis [77]. Natural killer (NK) cells are important regulators of innate and adaptive immunity and are closely linked to the regulation of cytotoxicity [78]. Experimental data shows NK cells can directly recognize the *Fusobacterium nucleatum* pathogen, leading to alveolar bone resorption and periodontitis [79]. The overactivity of NK is also purported to play a driving role in the progression of AD by producing a series of proinflammatory cytokines [80].

The findings of this *in silico* analysis must be considered in light of the strengths and limitations of this work. By using a machine learning-based feature selection method as the core technique, the most putatively robust crosstalk genes could be identified. Furthermore, functional molecular links were also analyzed in terms of differentially expressed pathways. The integrated analysis of multiple periodontitis-related GEO datasets enabled a larger sample size for improved accuracy of our computational prediction in the present study. The major limitation of the current approach is that no experimental validation of the identified pivotal genetic molecular linkage candidates was performed. This work has multiple implications for future research. Experimental and clinical studies focused on these candidates could be valuable from the perspectives of identification of shared susceptibility, exaggerating pathogenic mechanisms, biomarkers, and therapeutic targets relevant to precision medicine and drug development or repurposing.

## 5. Conclusion

Bioinformatic analysis integrating experimental transcriptomic data from Alzheimer's disease and periodontitis revealed the most robust potentially shared molecular linkages. Six crosstalk genes, C4A, C4B, CXCL12, FCGR3A, IL1B, and MMP3, three transcription factors, FOS, MEF2C, and USF2, and several pathways, JAK-STAT, MAPK, NF-kappa B, and natural killer cell-mediated cytotoxicity, emerged as top candidate shared molecular linkage entities and merit future research in experimental and clinical studies.

## Figures and Tables

**Figure 1:** Flowchart depicting study workflow.

**Figure 2:** Venn diagram showing the overlap between DEGs identified in the four periodontitis-related datasets.

**Figure 3:** Functional enrichment analysis of up- and downregulated periodontitis-related DEGs. (a) The functional terms (the biological processes (A) and KEGG pathways (B)) enriched by upregulated periodontitis-related DEGs. (b) The functional terms (the biological processes (A) and KEGG pathways (B)) enriched by downregulated periodontitis-related DEGs.

**Figure 4:** Protein-protein interaction (PPI) network associated with periodontitis. Red nodes represent the DEGs which were upregulated in periodontitis, green nodes represent the DEGs which were downregulated in periodontitis, and blue nodes represent other genes which were not DEGs but interacted with DEGs.

**Figure 5:** The crosstalk gene-related PPI network.

**Figure 6:** 48 crosstalk genes selected by using the Boruta algorithm (a) and 62 crosstalk genes selected by using the RFE algorithm (b).

**Figure 7:** The ROC curves of four periodontitis-related datasets.

**Figure 8:** The transcription factor-crosstalk gene target network.

**Figure 9:** Heatmaps depicting 137 signaling pathways enriched in the crosstalk genes in the four periodontitis-related datasets.

**Figure 10:** The crosstalk gene-differentially expressed pathway interaction network.

**Figure 11:** The ROC curves for 6 chronic periodontitis-related genes, C4A, C4B, CXCL12, FCGR3A, IL1B, and MMP3, in the four periodontitis-related datasets.

**Table 1:** Details of the included periodontitis-related GEO datasets.

Included four datasets	Type of periodontitis	Experimental platform	Number of examined genes	Number of inflamed gingival tissue samples	Number of healthy control samples	Number of total samples
GSE23586	3 patients with severe chronic periodontitis	GPL570	23,518	3	3	6
GSE16134	120 patients (65 with chronic periodontitis and 55 with aggressive periodontitis)	GPL570	24,441	241	69	310
GSE10334	63 with chronic periodontitis and 27 with aggressive periodontitis	GPL570	24,441	183	64	247
GSE79705	Generalized aggressive periodontitis (GAgP): *n* = 4; chronic periodontitis (CP): *n* = 4	GPL18734	19,305	8	4	12

**Table 2:** The number of up/downregulated DEGs identified in the four periodontitis-related datasets GSE23586, GSE16134, GSE10334, and GSE79705 at thresholds set for defining DEGs.

Data	Number of upregulated DEGs	Number of downregulated DEGs	Number of total DEGs	∣log2 FC∣	*p* value	Expression scale (if the data normalization was performed)
GSE23586	7	69	76	>1	<0.05	True
GSE16134	188	48	236	>1	<0.05	False
GSE10334	152	42	194	>1	<0.05	False
GSE79705	219	291	510	>0	<0.05	True

**Table 3:** Topological characteristics of the top 30 nodes in the periodontitis-related PPI network, ranked in descending order of degree.

Node	Label	Degree	Average shortest path length	Betweenness centrality	Closeness centrality	Clustering coefficient	Topological coefficient
MYC	DEG_down	1027	2.432727	0.177217	0.411061	0.001896	0.002805
HSPB1	DEG_down	433	2.638061	0.059908	0.379066	0.00278	0.005213
SMAD3	DEG_up	396	2.667636	0.052167	0.374864	0.004283	0.005425
UBC		395	2.112	0.241673	0.473485	0.004524	0.007004
TRIM27	DEG_up	334	2.864727	0.046792	0.349073	0.000791	0.006306
VIM	DEG_up	320	2.705212	0.037607	0.369657	0.005251	0.007619
YWHAH	DEG_up	282	2.838788	0.034115	0.352263	0.001868	0.00865
DDB1	DEG_down	276	2.76497	0.029677	0.361668	0.003531	0.008012
RPS3	DEG_down	275	2.844848	0.015036	0.351513	0.019323	0.014779
KAT5	DEG_down	245	2.717697	0.028224	0.367959	0.00716	0.007732
SMARCA4	DEG_down	242	2.715758	0.021646	0.368221	0.010116	0.008636
RPL13	DEG_down	234	2.755152	0.015773	0.362956	0.024541	0.011238
PLCG1	DEG_down	227	2.885091	0.030011	0.34661	0.002144	0.009614
FOS	DEG_up	226	2.880727	0.024538	0.347135	0.003265	0.009974
AP2M1	DEG_down	214	2.850182	0.025582	0.350855	0.007635	0.010848
SF3B3	DEG_down	203	2.765576	0.015188	0.361588	0.014583	0.010661
TP53RK	DEG_up	200	2.871394	0.013972	0.348263	0.01608	0.012798
MMS19	DEG_down	195	2.806909	0.022335	0.356264	0.004705	0.008763
RPS7	DEG_down	193	2.88303	0.008126	0.346857	0.028335	0.016367
MEPCE	DEG_down	189	2.905212	0.0145	0.344209	0.005066	0.012337
TUBB4B	DEG_down	173	2.880364	0.008167	0.347178	0.007595	0.019412
CDH1	DEG_down	171	2.888485	0.016186	0.346202	0.005848	0.011775
EZR	DEG_down	170	2.906667	0.016295	0.344037	0.004107	0.01554
DDX41	DEG_down	168	2.950061	0.009545	0.338976	0.007057	0.017509
NUDC	DEG_up	160	2.943758	0.016886	0.339702	0.00283	0.013954
SF3A2	DEG_down	156	2.949818	0.009075	0.339004	0.009926	0.01593
RPL27	DEG_down	147	2.912727	0.003949	0.343321	0.043985	0.020057
NIFK	DEG_up	145	3.107879	0.011111	0.321763	0.010345	0.016053
SRPRB	DEG_up	143	2.945333	0.017545	0.33952	0.001674	0.015983
ATP1A1	DEG_up	140	2.816606	0.011269	0.355037	0.009147	0.013032

**Table 4:** The 51 crosstalk genes that were upregulated and 41 crosstalk genes which were downregulated in periodontitis.

Regulation pattern in periodontitis	Crosstalk genes linking periodontitis and Alzheimer's disease
Upregulated	AMIGO1 (adhesion molecule with Ig-like domain 1; gene ID: 57463) ARG2 (arginase 2; gene ID: 384) BDKRB2 (bradykinin receptor B2; gene ID: 624) BRI3 (brain protein I3; gene ID: 25798) C1D (C1D nuclear receptor corepressor; gene ID: 10438) C3 (complement C3; gene ID: 718) C4A (complement C4A (Rodgers blood group); gene ID: 720) C4B (complement C4B; gene ID: 721) C4B_2 (complement component 4B (Chido blood group), copy 2; gene ID: 100293534) CASP7 (caspase 7; gene ID: 840) CD177 (CD177 molecule; gene ID: 57126) CD38 (CD38 molecule; gene ID: 952) CHCHD10 (coiled-coil-helix-coiled-coil-helix domain containing 10; gene ID: 400916) COX8A (cytochrome c oxidase subunit 8A; gene ID: 1351) CSF3 (colony-stimulating factor 3; gene ID: 1440) CTGF (cellular communication network factor 2; gene ID: 1490) CTSS (cathepsin S; gene ID: 1520) CXCL1 (C-X-C motif chemokine ligand 1; gene ID: 2919) CXCL12 (C-X-C motif chemokine ligand 12; gene ID: 6387) CXCL8 (C-X-C motif chemokine ligand 8; gene ID: 3576) CXCR4 (C-X-C motif chemokine receptor 4; gene ID: 7842) ENPP2 (ectonucleotide pyrophosphatase/phosphodiesterase 2; gene ID: 5168) FCGR3A (Fc fragment of IgG receptor IIIa; gene ID: 2214) FCGR3B (Fc fragment of IgG receptor IIIb; gene ID: 2215) FHL2 (four and a half LIM domains 2; gene ID: 2274) FOS (Fos proto-oncogene, AP-1 transcription factor subunit; gene ID: 2353) FOXO1 (forkhead box O1; gene ID: 2308) GSTK1 (glutathione S-transferase kappa 1; gene ID: 373156) GSTO1 (glutathione S-transferase omega 1; gene ID: 9446) HCLS1 (hematopoietic cell-specific Lyn substrate 1; gene ID: 3059) IGFBP7 (insulin-like growth factor binding protein 7; gene ID: 3490) IL1B (interleukin-1 beta; gene ID: 3553) LYZ (lysozyme; gene ID: 4069) MAK16 (MAK16 homolog; gene ID: 84549) MEF2C (myocyte-specific enhancer factor 2C; gene ID: 4208) MME (membrane metalloendopeptidase; gene ID: 4311) MMP1 (matrix metallopeptidase 1; gene ID: 4312) MMP3 (matrix metallopeptidase 3; gene ID: 4314) MS4A1 (membrane-spanning 4-domains A1; gene ID: 931) MSRA (methionine sulfoxide reductase A; gene ID: 4482) MZB1 (marginal zone B and B1 cell-specific protein; gene ID: 51237) NDUFB8 (NADH:ubiquinone oxidoreductase subunit B8; gene ID: 4714) PECAM1 (platelet endothelial cell adhesion molecule 1; gene ID: 5175) PLAT (plasminogen activator, tissue type; gene ID: 5327) PSENEN (presenilin enhancer, gamma-secretase subunit; gene ID: 55851) SEL1L (SEL1L adaptor subunit of ERAD E3 ubiquitin ligase; gene ID: 6400) SERPINI1 (serpin family I member 1; gene ID: 5274) ST6GAL1 (ST6 beta-galactoside alpha-2,6-sialyltransferase 1; gene ID: 6480) VCAN (versican; gene ID: 1462) VIM (vimentin; gene ID: 7431) WARS2 (tryptophanyl tRNA synthetase 2, mitochondrial; gene ID: 10352)

Downregulated	ABCA12 (ATP binding cassette subfamily A member 12; gene ID: 26154) ACE (angiotensin I converting enzyme; gene ID: 1636) ADRB1 (adrenoceptor beta 1; gene ID: 153) BCL2L2 (BCL2-like 2; gene ID: 599) BRSK1 (BR serine/threonine kinase 1; gene ID: 84446) CALML5 (calmodulin-like 5; gene ID: 51806) CALR (calreticulin; gene ID: 811) CD36 (CD36 molecule; gene ID: 948) CDH1 (cadherin 1; gene ID: 999) CDK5R1 (cyclin-dependent kinase 5 regulatory subunit 1; gene ID: 8851) CTDSP2 (CTD small phosphatase 2; gene ID: 10106) DNM1 (dynamin 1; gene ID: 1759) DSG1 (desmoglein 1; gene ID: 1828) FLG (filaggrin; gene ID: 2312) GJA1 (gap junction protein alpha 1; gene ID: 2697) GRHL3 (grainyhead-like transcription factor 3; gene ID: 57822) GRIN3B (glutamate ionotropic receptor NMDA type subunit 3B; gene ID: 116444) HM13 (histocompatibility minor 13; gene ID: 81502) HMGCR (3-hydroxy-3-methylglutaryl-CoA reductase; gene ID: 3156) HSPB1 (heat shock protein family B (small) member 1; gene ID: 3315) KAT5 (lysine acetyltransferase 5; gene ID: 10524) MAP3K12 (mitogen-activated protein kinase kinase kinase 12; gene ID: 7786) MED12 (mediator complex subunit 12; gene ID: 9968) MFN2 (mitofusin 2; gene ID: 9927) MYC (MYC proto-oncogene, bHLH transcription factor; gene ID: 4609) NEFL (neurofilament light; gene ID: 4747) NES (exportin 1; gene ID: 7514) NGF (nerve growth factor; gene ID: 4803) NOS3 (nitric oxide synthase 3; gene ID: 4846) NPTXR (neuronal pentraxin receptor; gene ID: 23467) PLXNA3 (plexin A3; gene ID: 55558) PPIL2 (peptidylprolyl isomerase-like 2; gene ID: 23759) PTGS1 (prostaglandin-endoperoxide synthase 1; gene ID: 5742) RPL13 (ribosomal protein L13; gene ID: 6137) SCIMP (SLP adaptor and CSK interacting membrane protein; gene ID: 388325) SPPL2B (signal peptide peptidase-like 2B; gene ID: 56928) TIAF1 (TGFB1-induced antiapoptotic factor 1; gene ID: 9220) TP73 (tumor protein P73; gene ID: 7161) TYRP1 (tyrosinase-related protein 1; gene ID: 7306) USF2 (upstream transcription factor 2, C-Fos interacting; gene ID: 7392) VEGFA (vascular endothelial growth factor A; gene ID: 7422)

**Table 5:** Topological characteristics of the top 30 nodes in the crosstalk gene-related PPI network, ranked in descending order of degree.

Node	Label	Degree	Average shortest path length	Betweenness centrality	Closeness centrality	Clustering coefficient	Topological coefficient
MYC	DEG_AD_down	1027	2.127525	0.466698	0.47003	5.03*E* − 04	0.001842
HSPB1	DEG_AD_down	433	2.36959	0.184598	0.422014	0.001636	0.003351
VIM	DEG_AD_up	320	2.663301	0.116611	0.375474	0.001763	0.005783
KAT5	DEG_AD_down	245	2.566359	0.089476	0.389657	0.003011	0.005621
RPL13	DEG_AD_down	234	2.589729	0.089708	0.386141	0.001394	0.005672
FOS	DEG_AD_up	226	2.883151	0.083642	0.346843	1.97*E* − 04	0.017606
CDH1	DEG_AD_down	171	2.93191	0.058428	0.341075	0	0.025911
TP73	DEG_AD_down	137	2.61483	0.046781	0.382434	0.006333	0.009173
FHL2	DEG_AD_up	136	2.641085	0.057192	0.378632	0.004031	0.00889
CALR	DEG_AD_down	135	2.812464	0.046142	0.35556	0.002764	0.010949
GSTK1	DEG_AD_up	111	2.988459	0.035152	0.334621	0	0.026289
MME	DEG_AD_up	104	2.836988	0.040386	0.352487	0.001307	0.011694
MED12	DEG_AD_down	91	2.695615	0.030682	0.370973	0.006105	0.012517
CASP7	DEG_AD_up	90	2.901039	0.027131	0.344704	0.005243	0.015603
DNM1	DEG_AD_down	84	2.960185	0.029086	0.337817	0.001147	0.023716
FOXO1	DEG_AD_up	67	2.977784	0.017403	0.33582	0.004071	0.026586
CXCR4	DEG_AD_up	65	2.998557	0.020851	0.333494	0.003846	0.028808
NOS3	DEG_AD_down	62	2.963647	0.018786	0.337422	0.002644	0.027957
NDUFB8	DEG_AD_up	56	3.042412	0.02136	0.328687	0	0.027447
UBC	Other gene	53	2.084824	0.149265	0.479657	0.015965	0.027336
NES	DEG_AD_down	53	2.920946	0.017012	0.342355	0.007983	0.022954
CDK5R1	DEG_AD_down	50	3.0176	0.0133	0.331389	0.002449	0.037222
NEFL	DEG_AD_down	49	2.913445	0.014886	0.343236	0.008503	0.024673
C3	DEG_AD_up	43	3.043278	0.01705	0.328593	0	0.042101
SEL1L	DEG_AD_up	42	3.036065	0.013066	0.329374	0	0.045635
DSG1	DEG_AD_down	41	3.046163	0.00857	0.328282	0	0.068464
GJA1	DEG_AD_down	41	3.035199	0.015703	0.329468	0	0.04037
MEF2C	DEG_AD_up	41	3.039238	0.008676	0.32903	0	0.068892
LYZ	DEG_AD_up	40	3.042123	0.008578	0.328718	0	0.065086
GSTO1	DEG_AD_up	38	2.820254	0.010905	0.354578	0.019915	0.030356

**Table 6:** Classification performance of the 48 feature selection-obtained crosstalk genes in the four periodontitis-related datasets.

	GSE16134			GSE10334			GSE23586			GSE79705		
	Samples: test set	Samples: SVM model predicts accurately	Accuracy	Samples: validation set	Samples: SVM model predicts accurately	Accuracy	Samples: validation set	Samples: SVM model predicts accurately	Accuracy	Samples: validation set	Samples: SVM model predicts accurately	Accuracy
Case	93	92	91.94%	183	177	88.26%	3	3	50%	8	8	66.66%
Control	31	22		64	41		3	0		4	0	
Total	124	114		247	218		6	3		12	8	

**Table 7:** Topological characteristics of the top 30 nodes in the TF-crosstalk gene target network, ranking in descending order.

Node	Label	Degree	Average shortest path length	Betweenness centrality	Closeness centrality	Clustering coefficient	Topological coefficient
FOS	DEG_up&TF	89	2.178295	0.206101	0.459075	0.020429	0.03825
VEGFA	DEG_down	77	2.211886	0.197219	0.452103	0.010936	0.038456
MEF2C	DEG_up&TF	76	2.328165	0.159945	0.429523	0.004211	0.044258
CDH1	DEG_down	69	2.540052	0.159392	0.393693	0	0.086634
CXCR4	DEG_up	47	2.596899	0.075105	0.385075	9.25*E* − 04	0.083836
MME	DEG_up	44	2.664083	0.04365	0.375364	0	0.131313
C4A	DEG_up	38	2.661499	0.029742	0.375728	0.01138	0.118617
VIM	DEG_up	38	2.521964	0.060293	0.396516	0.012802	0.065789
CSF3	DEG_up	36	2.550388	0.031734	0.392097	0.019048	0.075137
C4B	DEG_up	34	2.679587	0.018887	0.373192	0.012478	0.122037
VCAN	DEG_up	34	2.726098	0.030567	0.366825	0	0.143717
IL1B	DEG_up	33	2.741602	0.05746	0.36475	0	0.134602
BRSK1	DEG_down	30	2.741602	0.030404	0.36475	0	0.153788
SERPINI1	DEG_up	29	2.793282	0.019014	0.358002	0	0.127586
USF2	DEG_down&TF	27	2.591731	0.027575	0.385842	0.045584	0.081607
GRHL3	DEG_down	27	2.775194	0.027067	0.360335	0	0.150732
HSPB1	DEG_down	26	2.780362	0.017981	0.359665	0	0.155678
MMP3	DEG_up	26	2.607235	0.024377	0.383548	0.036923	0.074984
CTGF	DEG_up	25	2.788114	0.020669	0.358665	0	0.161905
HMGCR	DEG_down	25	2.767442	0.041119	0.361345	0	0.16
GATA2	TF	24	2.095607	0.052687	0.477189	0.018116	0.104678
PLAT	DEG_up	24	2.762274	0.028075	0.362021	0	0.173148
ETS1	TF	22	2.273902	0.03767	0.439773	0.012987	0.092022
NPTXR	DEG_down	22	2.826873	0.020478	0.353748	0	0.154545
AR	TF	21	2.24031	0.040698	0.446367	0.02381	0.105465
YBX1	TF	21	2.315245	0.037801	0.43192	0.004762	0.098928
BCL2L2	DEG_down	21	2.813953	0.018179	0.355372	0	0.144048
FCGR3A	DEG_up	21	2.81137	0.020521	0.355699	0	0.192799
ABCA12	DEG_down	20	2.79845	0.010961	0.357341	0	0.2
SP1	TF	20	2.191214	0.037362	0.456368	0.026316	0.109167
CDK5R1	DEG_down	20	2.824289	0.017878	0.354071	0	0.156098
FLG	DEG_down	20	2.653747	0.012281	0.376826	0.042105	0.093043

**Table 8:** The number of crosstalk gene-related DEPs within the four periodontitis-related datasets.

Data	Sample	DEP	DEP	DEP	Log FC	*p* value
		Up	Down	Total	Abs	
GSE23586	6	1	12	13	>1	<0.05
GSE16134	310	84	2	86	>1	<0.05
GSE10334	247	77	2	79	>1	<0.05
GSE79705	12	4	4	8	>0	<0.05

**Table 9:** The 12 overlapping genes between 48 feature selection-obtained crosstalk genes and periodontitis-related genes in the DisGeNET database. Among the 12 genes, 6 genes, C4A, C4B, CXCL12, FCGR3A, IL1B, and MMP3, were associated with chronic periodontitis.

Gene symbol	Gene ID	Disease ID	Disease name
C3	718	C0031099	Periodontitis
C4A	720	C0266929	Chronic periodontitis
C4B	721	C0266929	Chronic periodontitis
CXCL12	6387	C0266929	Chronic periodontitis
FCGR3A	2214	C0266929	Chronic periodontitis
FCGR3A	2214	C0031099	Periodontitis
FCGR3A	2214	C0031106	Periodontitis, juvenile
FCGR3A	2214	C0399447	Early-onset periodontitis
FCGR3A	2214	C0031030	Periapical periodontitis
FCGR3B	2215	C0399447	Early-onset periodontitis
FCGR3B	2215	C0031106	Periodontitis, juvenile
HSPB1	3315	C0031030	Periapical periodontitis
IL1B	3553	C1719494	Periodontitis, localized aggressive
IL1B	3553	C1719495	Aggressive periodontitis, generalized
IL1B	3553	C0399447	Early-onset periodontitis
IL1B	3553	C0001342	Acute periodontitis
IL1B	3553	C0031106	Periodontitis, juvenile
IL1B	3553	C0031030	Periapical periodontitis
IL1B	3553	C4025886	Severe periodontitis
IL1B	3553	C0031099	Periodontitis
IL1B	3553	C0266929	Chronic periodontitis
MME	4311	C0031099	Periodontitis
MMP3	4314	C0031106	Periodontitis, juvenile
MMP3	4314	C0001342	Acute periodontitis
MMP3	4314	C0266929	Chronic periodontitis
MMP3	4314	C0031099	Periodontitis
PLAT	5327	C1719495	Aggressive periodontitis, generalized
VEGFA	7422	C0031099	Periodontitis

## Data Availability

The data used to support the findings of this study are available from the corresponding author upon request.
